# The Efficacy of Immune Checkpoint Inhibitors vs. Chemotherapy for KRAS-Mutant or EGFR-Mutant Non-Small-Cell Lung Cancers: A Meta-Analysis Based on Randomized Controlled Trials

**DOI:** 10.1155/2022/2631852

**Published:** 2022-08-26

**Authors:** Wei Chen, Ling Li, Sheng Cheng, Junxian Yu

**Affiliations:** Department of Pharmacy, Beijing Friendship Hospital, Capital Medical University, Beijing, China

## Abstract

**Objective:**

To assess and compare the effectiveness of immune checkpoint inhibitors vs. chemotherapy for KRAS-mutant or EGFR-mutant non-small-cell lung cancers.

**Methods:**

Until February 19, 2022, Cochrane Library, PubMed, Web of Science, and Embase were searched for relevant randomized controlled trials (RCTs) in NSCLC. Progression-free survival (PFS) and overall survival (OS) were used as outcome measures. The studies were conducted using the Cochrane methodology for meta-analyses, and all statistical analyses were made with Review Manager Software (RevMan version 5.4).

**Results:**

Our meta-analysis included nine clinical trials including 5633 participants with NSCLC. Immune checkpoint drugs extended OS (hazard ratio (HR), 0.67; 95% confidence interval (CI), 0.60–0.76) and PFS (HR, 0.44; 95% CI, 0.35-0.56) in patients with EGFR wild-type compared to chemotherapy alone, whereas programmed cell death 1 ligand 1 (PD-L1)/programmed cell death-1 (PD-1) inhibitors with chemotherapy versus chemotherapy extended PFS in NSCLC patients with EGFR mutations (HR, 0.63; 95% CI, 0.42-0.94). Meanwhile, immune checkpoint inhibitors vs. chemotherapy improved the OS (HR, 0.65; 95% CI, 0.48–0.88) and PFS (HR, 0.49; 95% CI, 0.36–0.66) of NSCLC patients with KRAS mutation. NSCLCs with KRAS G12C mutation had a much better PFS with ICIs than with chemotherapy (HR, 0.38; 95% CI, 0.21–0.71).

**Conclusion:**

This research revealed that individuals with EGFR wild-type NSCLC or KRAS mutation may benefit from PD-L1/PD-1 inhibitors and that PD-L1/PD-1 inhibitors in combination with chemotherapy seem to be more successful than chemotherapy alone in NSCLC patients with EGFR mutation.

## 1. Background

Lung cancer is estimated to be the second most often diagnosed kind of cancer and the main reason of cancer mortality, accounting for about 2.2 million novel cases plus 1.8 million demises per year. NSCLC is the most prevalent subtype, accounting for 85% of all lung cancer occurrences [1]. While conventional chemotherapy, such as docetaxel, was authorized as a second-line therapy for progressive NSCLC, based on improved survival compared to optimal supportive care, its effectiveness is offset by significant adverse events [2]. With the advancement of immune checkpoint inhibitors (ICIs), they have become a more viable option for individuals with NSCLC [3]. Point mutations in the KRAS gene at sites 12 or 13 result in an amino acid substitution and RAS signaling pathway's constitutive activation. Additionally, this might interact with a variety of effectors, for example, phosphoinositide 3-kinase (PI3K) and transcription cascades' signal activator and transducer [4]. KRAS is the most frequently mutated oncogene in humans, with mutations occurring in up to 30% of individuals with NSCLC [5]. KRAS mutations are more prevalent in present or past smokers than in nonsmokers. Additionally, these mutations are very prevalent in smokers than nonsmokers (30% vs. 11%), as well as in Western than Asian inhabitants (26% vs. 11%) [6]. Although the successful use and marketing of small molecule inhibitors targeting the KRAS-G12C mutation in clinical trials has demonstrated that KRAS mutations can be successfully targeted, they are not yet used on a large scale in all countries [7, 8]. Therefore, according to current guidelines, ICI remains the best treatment for these patients [9]. In the great majority of instances, KRAS mutations are generally selective with anaplastic lymphoma kinase fusions and EGFR mutations, suggesting that KRAS mutations represent a discrete group of illness [10]. EGFR mutations are common in NSCLC and are clinically heterogeneous [11]. A small percentage of NSCLC patients with EGFR mutation respond well to treatment with appropriate molecularly targeted drugs and have fewer adverse effects [12]. However, for most patients with NSCLC whose tumors lack oncogenic driver modifications, targeted therapy is ineffective. Due to acquired drug resistance, essentially, all EGFR-mutant NSCLC patients inevitably develop drug resistance over time [13]. There are no further effective treatment options for NSCLC with disease progression due to the use of EGFR tyrosine kinase inhibitors (TKIs) [14].

However, the majority of clinical investigations omitted certain patients, for instance, people with mutations in the EGFR/KRAS gene. The evidence on the predictive significance of KRAS mutations in the NSCLC is inconsistent. There is a well-known meta-analysis that indicates that NSCLC patients with KRAS mutations had a worse survival rate (hazard ratio, 1.59; 95% CI: 1.16–1.56) [15]. However, in another meta-analysis, no significant prognostic impact of mutated KRAS on PFS (HR = 1.03; 95%CI) or on OS (HR = 1.10; 95%CI) was observed [16]. Following the research, we discovered that other meta-analyses contained incomplete genes or did not include a sufficient number of trials. To address these limitations, this meta-analysis sought to find studies examining the extent toward EGFR or KRAS or mutation status gives data on both the probability of a specific illness outcome from a very independent of treatment (prognostic factor) and possibility of advantage from a particular therapy (predictive factor) in NSCLC patients.

## 2. Materials and Methods

### 2.1. Literature Search

This meta-analysis and systematic review was conducted in compliance with the PRISMA guidelines on recommended reporting items for meta-analyses and systematic reviews [17]. A thorough search of PubMed, the Cochrane Library databases, Web of Science, and Embase was conducted in order to find all eligible trials with NSCLC from their inception through February 19, 2022, with no initiation date restriction.

We screen studies from PubMed database with “carcinoma, nonsmall cell lung”[MeSH Terms] AND (“PD-1”[All Fields] OR “pd-l1”[All Fields] OR (“pembrolizumab”[Supplementary Concept] OR “pembrolizumab”[All Fields]) OR (“nivolumab”[MeSH Terms] OR “nivolumab”[All Fields] OR “nivolumab s”[All Fields]) OR (“atezolizumab”[Supplementary Concept] OR “atezolizumab”[All Fields]) OR (“avelumab”[Supplementary Concept] OR “avelumab”[All Fields]) OR (“ipilimumab”[MeSH Terms] OR “ipilimumab”[All Fields]) OR (“tremelimumab”[Supplementary Concept] OR “tremelimumab”[All Fields]) OR (“durvalumab”[Supplementary Concept] OR “durvalumab”[All Fields])) AND (randomized clinical trial”[All Fields]).

### 2.2. Selection Criteria

The following primary criteria were used to determine inclusion:

1. The trial's primary objective should be NSCLC patients
2. Inhibitors of PD-L1/PD-1 must be included in the intervention
3. Chemotherapy should be administered to the control group
4. OS or PFS should be recorded for NSCLC patients with sensitive gene mutations (e.g., KRAS and EGFR).
5. Randomized controlled trials in Phase III or Phase II/III should be included only

The following criteria were used to exclude papers:

1. Editorials, observational studies, commentaries, and reviews were excluded
2. Abstracts and papers published in languages (e.g., Japanese and Chinese) other than English were excluded
3. Papers with inadequate data for evaluating the hazard risk of OS or PFS due to gene mutation

### 2.3. Data Extraction

All data for the study were retrieved and cross-checked separately by the two authors using a set of methods; discrepancies were addressed by conversation with the third author. The following data were collected: first author, trial phase, publication year, patient count, immunological target, control and experimental arms, treatment line, and HR for OS or PFS.

### 2.4. Study Quality's Assessment and Publication Bias

The bias' risk was evaluated in accordance with the Systematic Reviews of Interventions' Cochrane Handbook [18], which includes evaluating bias associated with concealment of allocation, random sequence generation, selective reporting of negative or/and positive findings, blinding, data integrity, and other sources of bias (OSB).

OSB were the following: explicit exclusion/inclusion criteria, any interest's conflict, and similar baseline data. All clinical trials used were registered. Additionally, the two researchers independently evaluated and verified the bias's risk; the findings were cross-checked, and any differences were fixed by consultation with the third researcher.

### 2.5. Statistical Analysis

Our systematic review, which included the making of forest plots, was conducted with the help of Review Manager (version 5.4; Cochrane Collaboration). The effect sizes were calculated using the CI and the HR. If *p* value for heterogeneity was <0.10 or *I*^2^ was more than 50% in this analysis, the null hypothesis of the study that the trials were homogeneous would be rejected. If there was considerable heterogeneity in the findings of the included studies, summary estimate was measured using the random effects model [19]. Unless otherwise specified, the summary estimates will be established on the fixed-effects model (FEM). Also, it was calculated using the inverse variance approach, assuming that the included trials had similar effect sizes. A funnel plot was utilized to demonstrate publication bias.

## 3. Results

### 3.1. Literature Search Results

A total of 804 potentially related articles were uncovered by our search approach in databases. After duplicates, screened titles and abstracts were excluded, and 15 articles remained for further evaluation. After a full article review was conducted, 9 separate trials were incorporated.  Figure 1 illustrates our selection method and the reasons for study exclusion.

### 3.2. Characteristics of the Selected Articles

Table 1 summarizes the RCTs' features. Our meta-analysis included nine clinical trials including 5633 participants with NSCLC. Each clinical trial was a randomized controlled Phase II/III trial. Five of these trials used first-line treatment, while four used second- or additional-line therapy. Six studies including PD-1 inhibitors (two involving nivolumab and 4 involving pembrolizumab) and three involving PD-L1 inhibitors were identified (all with atezolizumab).

Seven trials assessed the effectiveness of ICIs in NSCLC patients who were wild-type or had an EGFR mutation (three with hazard rate of OS and three with hazard rate of PFS) [20–26]. Five trials examined the impact of PD-L1 or PD-1 inhibitors in patients with NSCLC who had a KRAS mutation or were wild-type (four with hazard rate of OS and three with hazard rate of PFS) [21, 25–28].

### 3.3. Study Quality's Evaluation and Publication Bias

Because of the complexity inherent in the course of concealing allocation, some of the integrated studies exhibited a high [25, 26] or uncertain risk [20, 21, 24] of selection bias. Each of them included a rather comprehensive summary of the result data illustrates the risk assessment process for bias (Figures 2 and 3). Little publication bias was observed in reports evaluating EGFR mutations and KRAS mutations, and the funnel plots are shown in Figures 4 and 5.

### 3.4. Wild-Type or EGFR Mutation

Four RCTs examined the OS for NSCLC patients with/without EGFR mutations [21–23, 25]. There was little variability in OS analysis for the EGFR mutation (*I*^2^ = 0%). As a result, a FEM was adopted in this investigation. According to the meta-analysis, as shown by Figure 6, ICIs were as effective as chemotherapy in handling NSCLC patients with EGFR mutations for OS (HR, 1.11; 95% CI, (0.80, 1.53)). In the overall (*I*^2^ = 0%) study of EGFR wild-type, there was still a modest degree of heterogeneity. As a result, our investigation used the fixed-effects model. The meta-analysis revealed (Figure 6) that ICIs vs. chemotherapy considerably enhanced the OS of NSCLC patients with EGFR wild-type (HR, 0.67; 95% CI, (0.60, 0.76)). ICIs seemed to have a significantly greater effectiveness than chemotherapy alone in individuals with EGFR wild-type NSCLCs than in those with EGFR mutations (*χ*^2^ = 8.11; *p* = 0.004). OS superior to chemotherapy with ICIS in EGFR genetically tested NSCLC patients (HR, 0.71; 95% CI, (0.64, 0.80)).

Three RCTs examined the PFS for NSCLC patients with/without EGFR mutations [20, 24, 26]. There was little variability in PFS analyses for EGFR mutations (*I*^2^ = 0%). The meta-analysis demonstrated (Figure 7) that PD-L1/PD-1 inhibitors in conjunction with chemotherapy vs. chemotherapy significantly improved the PFS of NSCLC patients with EGFR mutations (HR, 0.63; 95% CI, (0.42, 0.94)). There was moderate heterogeneity in the entire (*I*^2^ = 57%) study of EGFR wild-type. According to the meta-analysis (Figure 7), immune checkpoint drugs vs. chemotherapy extended the PFS of NSCLC patients with EGFR wild-type (HR, 0.44; 95% CI, (0.35, 0.56)). There was also an insignificant difference in PFS between patients with EGFR mutations and those with wild-type EGFR NSCLCs (*χ*^2^ = 2.3 ; *p* = 0.13). Treatment with ICIs is more effective than chemotherapy in this subset of the population (HR, 0.48; 95% CI, (0.39, 0.60)).

### 3.5. Wild-Type or KRAS Mutation

There were four RCTs that compared OS for NSCLC with or without the KRAS mutation [21, 25, 27, 28]. OS analysis revealed modest heterogeneity for the KRAS mutation (*I*^2^ = 29%). As a result, our investigation used a FEM. The meta-analysis revealed that ICIs vs. chemotherapy improved OS in NSCLC patients with KRAS mutations (HR, 0.65; 95% CI, (0.48, 0.88)), as shown by Figure 8. There was little variability in OS analysis for KRAS wild-type (*I*^2^ = 0%). As a result, the fixed-effects model was utilized in this research as well. As shown by Figure 8, the meta-analysis further revealed that there was, also, no significant difference in OS between immune checkpoint inhibitors and chemotherapy for NSCLC patients with KRAS wild-type (HR, 0.9; 95% CI, 0.71–1.16). Anti-PD-L1 treatment seemed to be substantially more effective than chemotherapy in patients with KRAS-mutated NSCLCs than with KRAS wild-type (*χ*^2^ = 2.8 ; *p* = 0.09). Treatment with ICIs produced much better results than chemotherapy in this group (HR, 0.79; 95% CI, 0.65–0.96).

Three RCTs examined the PFS of NSCLC patients with/without the KRAS mutation [26–28]. There was little variability in PFS analyses for KRAS mutations (*I*^2^ = 0%). The meta-analysis demonstrated (Figure 9) that ICIs were more effective than chemotherapy in extending the PFS of NSCLC patients with KRAS mutations (HR, 0.49; 95% CI, 0.36–0.66). For KRAS wild-type, PFS analysis revealed a significant degree of heterogeneity (*I*^2^ = 94%). According to Figure 9, KRAS wild-type NSCLCs treated with ICIs have improved PFS compared to chemotherapy (HR, 0.68; 95% CI, 0.54–0.84).

NSCLCs with KRAS mutations have an overall advantage over KRAS wild-type in PFS (*χ*^2^ = 2.86 ; *p* = 0.09). PFS of ICI treatment is superior to chemotherapy in a population of NSCLC patients tested for KRAS genes (HR, 0.61; 95% CI, 0.51–0.72).

Two RCTs examined the PFS of NSCLC patients with KRAS G12C mutation [26, 28]. There was little variability in PFS analyses for KRAS G12C mutations (*I*^2^ = 0%).  Figure 10 shows that NSCLC patients with KRAS G12C mutation had a much better PFS with ICIs than with chemotherapy (HR, 0.38; 95% CI, 0.21–0.71).

## 4. Discussion

Our research indicates that PD-L1 inhibitors had more effectiveness than chemotherapy in extending the survival of NSCLC patients with KRAS mutations. Additionally, it demonstrated that KRAS-mutant NSCLC gained more benefit from treatment with ICIs than KRAS wild-type. Among KRAS G12C-mutated NSCLCs, the efficacy of treatment with ICIs was better than the mean of KRAS mutation (HR, 0.38; 95% CI, 0.21–0.71 vs. HR, 0.49; 95% CI, 0.36–0.66). In NSCLC, KRAS oncogene substitutions often occur at codons 12 and 13 of exon 2, and common codon variants include G12C, G12D, G12V, and G12A [29, 30]. Of note, it has been shown that NSCLC with G12C, G12V, and G12A mutations are typical of smoking-associated tumors with high tumor mutation burden (TMB), with the exception of the KRAS-G12D point mutation [31, 32]. In never smokers, the most common KRAS mutation is KRAS-G12D [33]. A recent study has shown that a high TMB value indicates chromosomal instability that results in increased neoantigen generation and immune cell recruitment, and elevated TMB further increases the likelihood of ICI benefit [34, 35]. This implies that G12C, G12V, and G12A mutations are associated with biomarkers that predict benefit from ICIs, whereas G12D mutations lead to poor prognosis in NSCLC patients treated with ICIs. This is consistent with Aredo et al.'s study, and our meta-analysis also showed that G12C mutations improved the benefit of ICIs [36]. Analyzed from another perspective, PD-L1 inhibitors are more effective than chemotherapy for patients with high PD-1 expression [37]. The results of 23 studies revealed that patients with KRAS-mutant NSCLC were much more expected to be PD-L1 positive than patients with KRAS wild-type tumors (odd ratio = 1.87; 95% CI, (1.34, 2.61); *p* = 0.0002), indicating a significant positive association between PD-L1 expression and KRAS mutation status [38]. This is a possible explanation for our findings. On tumor cells, PD-L1 expression may be upregulated in response to a T-cell response or can be produced through oncogenic signaling [39]. As a result, cancers with KRAS mutation had a higher level of T-cell infiltration than tumors with KRAS wild-type. Taken together, these findings may help explain how KRAS mutations are amenable to immunotherapy.

Our meta-analysis indicates that the lack of benefit from single-agent PD-1/PD-L1 inhibitors (HR, 1.11; 95% CI, (0.80, 1.53)) compared to chemotherapy in patients with NSCLC who had an EGFR mutation might well be partly explained by reduced PD-L1 expression. What is more intriguing is that PD-L1 or PD-1 inhibitors in combination with chemotherapy seem to be more successful (PFS of 0.63; 95% CI, 0.42-0.94) in NSCLC patients who had an EGFR mutation. It was similar to previous meta-analysis (OS of 0.66; 95% CI, 0.40–1.00), but fewer randomized controlled trials were included, and further data would be required in the future to support it [40]. Meanwhile, our study indicated that individuals with EGFR wild-type NSCLC may benefit from PD-1/PD-L1 inhibitors in terms of PFS and OS. The most frequency point mutation for EGFR is 18, 19, 20, and 21 [41]. One research showed poor clinical benefit of ICIs in patients with EGFR 19 mutations [42]. Another study showed that ICIs were more effective than 19 DEL patients compared to EGFR 21 L858R patients [43]. In addition, EGFR 21 L858R subtypes tend to have high PDL1 expression and higher TMB. This suggests that EGFR 21 L858R subtypes may benefit from treatment with ICIs. The IMMUNOTARGET registry study reported that EGFR 20 T790M patients had the shortest PFS compared to other EGFR-mutant subtypes [44]. EGFR 18 G719 has high TMB, and its OS is also higher than other EGFR subgroups [45]. This also suggests that EGFR 18 G719 may benefit from ICI treatment. Our data suggest that EGFR and KRAS mutations may be used as possible predictive variables for anti-PD-1/PD-L1 treatment in patients with NSCLC. These possible prognostic indicators may assist NSCLC patients in pursuing more personalized treatment choices.

Our research, however, includes the following drawbacks. To begin, it was based on public data rather than on individual patient data, reducing its internal validity. Second, since not all of the participants had EGFR or KRAS mutation detection findings, the quantity of patient information on EGFR or KRAS mutations that we have access to is insufficient. Finally, PFS may not be an adequate effectiveness metric owing to the action's mechanism of PD-L1 and PD-1 inhibitors, which may have consequences in pseudoprogression because of inflammatory cell infiltration to the tumor site [46]. As a consequence, PFS data should be read cautiously when comparing PD-L1 and PD-1 inhibitors.

Future research should focus on the effect of different loci of KRAS, EGFR, or BRAF mutations on the therapeutic effect of ICIs, not just mutant or wild-type. Additionally, the mechanism of linkage between these gene alterations should be investigated further for improved clinical use.

## 5. Conclusion

In summary, our research demonstrates that patients with KRAS mutations or EGFR wild-type NSCLC may benefit from PD-1/PD-L1 inhibitors and that PD-1/PD-L1 inhibitors in combination with chemotherapy seem to be more successful than chemotherapy alone in NSCLC patients with EGFR mutations. NSCLCs with KRAS G12C mutation significantly benefit from treatment with ICIs.

## Figures and Tables

**Figure 1:** Flow diagram depicting the process of searching for and selecting relevant literature. The research followed the PRISMA 2020 statement: an updated standard for systematic review reporting. OS: overall survival; PFS: progression-free survival.

**Figure 2:** The bias' risk summary; green: low risk of bias, yellow: unclear risk of bias, and red: high risk of bias.

**Figure 3:** The bias' risk graph.

**Figure 4:** Evaluation of funnel plots for EGFR mutations.

**Figure 5:** Evaluation of funnel plots for KRAS mutations.

**Figure 6:** Forest plot for OS of NSCLC patients with wild-type or EGFR mutation.

**Figure 7:** Forest plot for PFS in patients with NSCLC who had the wild-type or EGFR mutation.

**Figure 8:** Forest plot for OS of NSCLC patients with KRAS mutation or wild-type.

**Figure 9:** Forest plot for PFS of NSCLC patients with the wild-type or KRAS mutation.

**Figure 10:** Forest plot for PFS of NSCLC patients with the KRAS-G12C mutation.

**Table 1:** Characteristics of the studies included in the meta-analysis.

Study	Clinical trials	Phase	Patients	Immune target	Experimental arms	Control arms	Therapeutic line	Primary outcome
Rittmeyer et al. (2016)	OAK	III	850	PD-L1	Atezolizumab	Docetaxel	>1	OS
Borghaei et al. (2015)	CHECKMATE 057	III	582	PD-1	Nivolumab	Docetaxel	>1	OS
Fehrenbacher et al. (2016)	POPLAR	II	287	PD-L1	Atezolizumab	Docetaxel	>1	OS
Socinski et al. (2018)	IMPOWER150	III	692	PD-L1	Atezolizumab+BCP	BCP	1	PFS
Arrieta et al. (2020)	PROLUNG	II	78	PD-1	Pembrolizumab+docetaxel	Docetaxel	1	PFS
Patel et al. (2020)	PACIFIC	III	713	PD-1	Pembrolizumab+docetaxel	Docetaxel	1	PFS
Herbst et al. (2019)	KEYNOTE-042	II	782	PD-1	Pembrolizumab	Docetaxel	1	OS, PFS
Herbst et al. (2016)	KEYNOTE-010	II/III	1033	PD-1	Nivolumab	Docetaxel	>1	OS
Gadgeel et al. (2019)	KEYNOTE-189	II	616	PD-1	Pembrolizumab+docetaxel	Docetaxel	1	OS, PFS

BCP: bevacizumab plus carboplatin plus paclitaxel.

## Data Availability

This meta-analysis and systematic review was conducted in compliance with the PRISMA guidelines on recommended reporting items for meta-analyses and systematic reviews. A thorough search of PubMed, the Cochrane Library databases, Web of Science, and Embase was conducted in order to find all eligible trials with NSCLC from their inception through February 19, 2022, with no initiation date restriction. We screen studies from the PubMed database with “carcinoma, nonsmall cell lung”[MeSH Terms] and (“PD-1”[All Fields] or “pd-l1”[All Fields] OR (“pembrolizumab”[Supplementary Concept] OR “pembrolizumab”[All Fields]) OR (“nivolumab”[MeSH Terms] OR “nivolumab”[All Fields] OR “nivolumab s”[All Fields]) OR (“atezolizumab”[Supplementary Concept] OR “atezolizumab”[All Fields]) OR (“avelumab”[Supplementary Concept] OR “avelumab”[All Fields]) OR (“ipilimumab”[MeSH Terms] OR “ipilimumab”[All Fields]) OR (“tremelimumab”[Supplementary Concept] OR “tremelimumab”[All Fields]) OR (“durvalumab”[Supplementary Concept] OR “durvalumab”[All Fields])) AND (randomized clinical trial”[All Fields]).

## Abbreviations

EGFR: Epidermal growth factor receptor
NSCLC: Non-small-cell lung cancer
RCTs: Randomized controlled trials
PFS: Progression-free survival
OS: Overall survival
HR: Hazard ratio
CI: Confidence interval
PD-L1: Programmed cell death ligand 1
PD-1: Programmed cell death-1
ICIs: Immune checkpoint inhibitors
PI3K: Phosphoinositide 3-kinase
OSB: Other sources of bias
FEM: Fixed-effects model
TMB: Tumor mutation burden.
